The article "Synergistic Apoptosis of CML Cells by Buthionine Sulfoximine and Hydroxychavicol Correlates with Activation of AIF and GSH-ROS-JNK-ERK-iNOS Pathway" was retracted in 2025. Reasons: errors in the data; errors in the images; duplicated images; duplicated data.

# Synergistic Apoptosis of CML Cells by Buthionine Sulfoximine and Hydroxychavicol Correlates with Activation of AIF and GSH-ROS-JNK-ERK-iNOS Pathway

**DOI:** 10.1371/journal.pone.0073672

**Published:** 2013-09-09

**Authors:** Avik Acharya Chowdhury, Jaydeep Chaudhuri, Nabendu Biswas, Anirban Manna, Saurav Chatterjee, Sanjit K. Mahato, Utpal Chaudhuri, Parasuraman Jaisankar, Santu Bandyopadhyay

**Affiliations:** 1 Division of Cancer Biology and Inflammatory Disorder, Council of Scientific and Industrial Research (CSIR)-Indian Institute of Chemical Biology (IICB), Kolkata, India; 2 Division of Chemistry, CSIR-IICB, Kolkata, India; 3 The Institute of Hematology and Transfusion Medicine, Medical College, Kolkata, India; University of California, Merced, United States of America

## Abstract

**Background:**

Hydroxychavicol (HCH), a constituent of Piper betle leaf has been reported to exert anti-leukemic activity through induction of reactive oxygen species (ROS). The aim of the study is to optimize the oxidative stress –induced chronic myeloid leukemic (CML) cell death by combining glutathione synthesis inhibitor, buthionine sulfoximine (BSO) with HCH and studying the underlying mechanism.

**Materials and Methods:**

Anti-proliferative activity of BSO and HCH alone or in combination against a number of leukemic (K562, KCL22, KU812, U937, Molt4), non-leukemic (A549, MIA-PaCa2, PC-3, HepG2) cancer cell lines and normal cell lines (NIH3T3, Vero) was measured by MTT assay. Apoptotic activity in CML cell line K562 was detected by flow cytometry (FCM) after staining with annexinV-FITC/propidium iodide (PI), detection of reduced mitochondrial membrane potential after staining with JC-1, cleavage of caspase- 3 and poly (ADP)-ribose polymerase proteins by western blot analysis and translocation of apoptosis inducing factor (AIF) by confocal microscopy. Intracellular reduced glutathione (GSH) was measured by colorimetric assay using GSH assay kit. 2′,7′-dichlorodihydrofluorescein diacetate (DCF-DA) and 4-amino-5-methylamino-2′,7′-difluorofluorescein (DAF-FM) were used as probes to measure intracellular increase in ROS and nitric oxide (NO) levels respectively. Multiple techniques like siRNA transfection and pharmacological inhibition were used to understand the mechanisms of action.

**Results:**

Non-apoptotic concentrations of BSO significantly potentiated HCH-induced apoptosis in K562 cells. BSO potentiated apoptosis-inducing activity of HCH in CML cells by caspase-dependent as well as caspase-independent but apoptosis inducing factor (AIF)-dependent manner. Enhanced depletion of intracellular GSH induced by combined treatment correlated with induction of ROS. Activation of ROS- dependent JNK played a crucial role in ERK1/2 activation which subsequently induced the expression of inducible nitric oxide synthase (iNOS). iNOS- mediated production of NO was identified as an effector molecule causing apoptosis of CML cells.

**Conclusion/Significance:**

BSO synergizes with HCH in inducing apoptosis of CML cells through the GSH-ROS-JNK-ERK-iNOS pathway.

## Introduction

Glutathione (GSH) is the major cellular antioxidant system which maintains the redox balance in cells. The important redox modulating enzymes like thiol reductases, peroxiredoxins and peroxidases depend on the pool of GSH. Therefore, strategies to induce a depletion of the GSH pool could have a profound effect on cell survival and drug sensitivity by altering the cells’ redox balance. It is reported that phenyl ethyle isothiocyanate (PEITC), sulforaphane cause a depletion of GSH pool and subsequent cell death [1], [2]. Depletion of GSH pool can also be achieved by inhibiting its synthesis. Buthionine sulphoximine (BSO) is most effective which is an inhibitor of glutamylcysteine synthetase (γ-GCS), the rate-limiting enzyme for GSH synthesis [3], [4]. This compound has been shown to cause GSH depletion and exhibits enhanced chemotherapeutic activity of different anti-cancer drugs [5], [6]. Recent reports suggest that BSO sensitizes antihormone- resistant breast cancer cells to estradiol treatment [7], [8]. Antimony-trioxide- and arsenic-trioxide-induced apoptosis in myelogenic and lymphatic cell lines is enhanced by BSO [9]. Enhanced anti-leukemic activity is also seen in combination treatment of BSO and Kanamycin F [10].

Hydroxychavicol (HCH), a phenolic compound of Piper betle leaves has anti-mutagenic and anti-carcinogenic activity [11], [12]. Antimicrobial, antioxidant and anti-inflammatory properties were also attributed to HCH [13]. Recent literature suggests that HCH has potential to eliminate prostate cancer cells [14]. Studies also suggested apoptosis of oral carcinoma cells by HCH through induction of reactive oxygen species (ROS) [15]. Our previous finding showed that HCH induces apoptosis in CML cells by ROS- mediated pathway [16]. Despite production of high level of ROS, HCH does not aggravate the depletion of intracellular GSH at moderate concentration [15], [16]. In view of this, we examined the potential effect of BSO to augment the anti-cancer effect of HCH in CML cells and investigate the possible mechanisms of cell death and apoptosis.

Another important aspect of HCH-induced apoptosis is the signaling by mitogen-activated protein kinases (MAPKs) [16]. It is generally accepted that the stress-activated protein kinase c-Jun NH2-terminal kinase (JNK) and the p38 kinase are associated to apoptosis induction, while the extracellular signal regulated protein kinases (ERK) behave as survival factor [17], [18]. Emerging studies revealed that ERK not only contribute to cell survival but under certain situations aberrant ERK activation can promote cell death [19], [20], [21]. JNK inhibition was also reported to potentiate apoptosis in some cell models [22], [23]. MAPK signaling pathways have been considered to be promising targets for antitumor therapy [24] and the crosstalk among these pathways within the cancer cells is complex [25], [26].

In the present report we analyzed the effects of GSH depletion on MAPK pathway. The results indicate that JNK positively activated ERK in BSO plus HCH-induced apoptosis in CML cells and this effect is mediated by early depletion of GSH. The combination of low concentration of HCH and BSO synergistically induced apoptosis in K562 cells through a JNK-ERK1/2-iNOS-mediated pathway.

## Materials and Methods

### Ethics Statement

Fresh peripheral blood samples from three CML patients were collected from Institute of Haematology and Transfusion Medicine, Medical College, Kolkata. Written informed consent according to the Declaration of Helsinki was obtained from all patients with prior approval from The Internal Review Board of Indian Institute of Chemical Biology, Kolkata, India. The Institutional Review Board approved this study.

### Cell Lines and Culture

CML cell line K562, acute T-lymphoblastic cell line Molt 4 and histiocytic lymphoblastic cell line U937, lung adenocarcinoma cell line A549, pancreatic adenocarcinoma cell line MIA-PaCa2, hepatic carcinoma cell line HepG2 and prostate cancer cell line PC-3 were purchased from the American Type Culture Collection (Manassas, VA). Normal cell lines NIH3T3 and Vero were purchased from National Centre for Cell Science, Pune, India. Other CML cell lines KU812 [27] and KCL22 [28] were generously provided by Dr. Carlo Gambacorti-Passerini (Instituto Nazionale Tumori, Milan, Italy). K562, Molt 4, U937, KU812, KCL22, MIA-PaCa2 and PC-3 were maintained in RPMI-1640 containing 10% fetal bovine serum (FBS), 100 U/ml penicillin and 100 µg/ml streptomycin (Life Technologies, New Delhi, India). A549, HepG2, NIH3T3 and Vero were cultured in DMEM medium containing 10% FBS, 100 U/ml penicillin with 100 µg/ml streptomycin.

Fresh peripheral blood sample was also collected from a normal donor. Mononuclear cells were separated by Histopaque (Sigma-Aldrich, St. Louis, MO, USA) density gradient centrifugation.

### Reagents and Antibodies

Hydroxychavicol (HCH) was purified as previously described [16]. BSO was purchased from MP Biomedicals (Santa Ana, CA, USA). The p38 inhibitor SB203580,extracellular signal regulated kinase 1/2 (ERK1/2) inhibitor PD98059, JNK inhibitor SP600125, 2′,7′-dichlorodihydrofluorescein diacetate (DCF-DA),4-amino-5-methylamino-2′,7′-difluorofluorescein (DAF-FM), 2–4 carboxyphenyl-4,4,5,5-tetramethylimidazoline-1-oxyl-3-oxide (c-PTIO), glutathione monoethyle ester (GME), JC-1, Z-VAD-FMK, Z-IETD-FMK and LEHD-CHO were obtained from Calbiochem (San Diego, CA, USA). Antibodies to cleaved-caspase 3, cleaved caspase 9, cleaved caspase-8, cleaved- poly (ADP-ribose) polymerase (PARP), endothelial nitric oxide synthase (eNOS), phospho-eNOS (Ser1177), neuronal nitric oxide synthase (nNOS) and phospho p38 (Thr180/Tyr182) were purchased from BD Biosciences (San Jose, CA, USA). Antibodies to phospho ERK1/2, ERK, phospho JNK, JNK, p38, inducible nitric oxide synthase (iNOS), Cox4, Cytochrome c and Actin were from Santa Cruz Biotechnology (Santa Cruz, CA, USA). Antibody to phospho-nNOS (Ser1417) was from Upstate (Billerica, MA, USA).

### Cell Viability and Apoptosis Assays

MTT assay was performed to determine cell viability. Cells were seeded in 96-well plates at cell density 10^4^/well, treated with HCH or BSO or in combination and incubated at 37°C in 5% (v/v) CO_2_ for indicated times. Viable cell numbers were determined by tetrazolium salt conversion to its formazan dye and absorbance was measured at 550 nm. Viability of primary CML cells was determined by trypan blue dye exclusion assay.

For determination of apoptotic cells, cells were seeded at 1.0×10^5^ cells in 24 well plates. Apoptosis was measured after indicated treatment using annexin V-fluorescein isothiocyanate (AnnexinV-FITC) and propidium iodide (PI). Analysis was done in a flow cytometer (BD FACSAria, Becton–Dickinson, San Jose, CA).

### Measurement of Intracellular Hydrogen Peroxide

For measurement of intracellular H_2_O_2_, control and treated K562 cells were incubated for 20 min at 37°C with 10 µM DCF-DA, washed with PBS and analyzed in a flow cytometer.

### Measurement of Intracellular Nitric Oxide

For measurement of intracellular nitric oxide (NO), treated and untreated cells were incubated with the cell permeable dye DAF-FM (3 µM) for 45 min at 37°C. Cells were washed with PBS and analyzed in a flow cytometer.

### Mitochondrial Membrane Permeability Assay

BSO plus HCH treated or untreated cells (1×10^5^) were incubated with mitochondrial membrane potential sensitive dye JC-1 (5 µM) for 15 min at room temperature in dark and analyzed by flow cytometry.

### Measurement of Intracellular GSH

Intracellular GSH contents were measured using a Glutathione Assay kit (Cayman, Michigan, USA). In brief, 2×10^6^ cells were sonicated in 5% metaphosphoric acid. Particulate matters were separated by centrifugation at 10000×g at 4°C. The supernatant were used for the intracellular GSH measurement as per manufacturer’s protocol.

### Confocal Microscopy

K562 cells were exposed either to indicated concentration of BSO or HCH alone or in combination in the presence or absence of indicated inhibitor for 18 h. Cells were collected by centrifugation, washed with PBS. After fixation with 4% paraformaldehyde for 30 min at room temperature, cells were permeabilized with 1% Triton X-100 (Sigma–Aldrich) for 5 min. These cells were then blocked in 1% bovine serum albumin solution for 30 min. The cells were incubated with rabbit anti-AIF primary antibody (Santa Cruz Biotechnology) for 45 min at room temperature. After washing with PBS cells were incubated with PE conjugated goat anti-rabbit secondary antibody (BD Biosciences) for 45 min at room temperature. Cell nuclei were stained with 4′,6-diamidino-2-phenylindole (DAPI) (Calbiochem). The slides were imaged in a Nikon A1R confocal microscope (Nikon, Tokyo, Japan).

### Sub-cellular Fractionation

The mitochondrial and cytoplasmic fractions of K562 cells were separated by ProteoExtract Cytosol/Mitochondria Fractionation Kit (Calbiochem), as per manufacturer’s protocol.

### Western Blot Analysis

After treatment as indicated, cells were collected by centrifugation, and lysed by sonication using RIPA buffer. 40 µg total cellular proteins were separated by SDS–polyacrylamide gel electrophoresis (PAGE) containing 10%–12% polyacrylamide, transferred to PVDF membrane and probed with primary antibodies followed by horseradish peroxidase-conjugated secondary antibody. Blots were developed by chemiluminescence method using Amersham ECL+ chemiluminescence kit.

### siRNA Transfections

Cells were transfected with control siRNA or indicated siRNAs (purchased from Dharmacon Inc., Lafayette, CO, USA) as described in respective figure legends. Transfections were carried out following the manufacturer’s instructions. The siRNA transfection reagent was also purchased from Dharmacon. 48 hour post-transfection, cells were treated with BSO or HCH or in combination as indicated.

### Statistical Analysis

Statistical analyses were performed using Student’s t-test.

The software CalcuSyn (BIOSOFT®, Cambridge, UK) was used to analyze dose effect relationship by the Monte-Carlo method. The combination index (CI) evaluated for K562 cells and hPBMC treated with BSO (25 µM, 50 µM, 100 µM) and HCH (5 µM, 10 µM, 20 µM) alone or in combination. The effects were entered as the input for CalcuSyn analysis as a constant ratio combination and the combination index (CI) value were recorded. The drug treatment was assessed based on the table for describing synergism or antagonism with the CI method. CI values less than 1.0 indicate synergism, CI values equal to 1.0 indicate additive effect, and CI values more than 1.0 indicate an antagonistic effect.

## Results

### Combination of HCH and BSO Induces Preferential Cytotoxicity Towards Leukemic Cell Lines Compared to Other Cancer Cell Lines and Normal Cells

We recently reported that HCH possesses anti-leukemic property with IC50 value more than 20.0 µM [16], [29]. HCH-induced ROS plays an important role for its anticancer activity [16]. BSO is known for its potential to deplete intracellular GSH. We therefore investigated the combination of these two molecules on the cytotoxic effect on a number of cancerous and non-cancerous cell lines. Initially, CML cell line K562 was treated with different concentrations of HCH or BSO for evaluation of cytotoxicity by MTT assay. As expected, IC50 of HCH on K562 cells was 20.0±10.0 µM (Fig. 1A). In contrast, BSO showed marginal cytotoxicity at concentrations more than 1 mM (Fig. 1A). Of interest, combination of these two molecules at much lower concentrations induced drastic cytotoxicity in K562 cells (Fig. 1B). The lowest concentration of HCH and BSO for the synergistic effect was 5 µM and 25 µM respectively. Next we evaluated the effect of this combination on a number of leukemic cell lines [two CML cell lines (KCL22, KU812), one T lymphoblastic leukemia cell line (Molt-4), acute myeloid leukemia cell line (U937) (Fig. 1C)], non-leukemic cancer cell lines [lung adenocarcinoma (A549), pancreatic cancer (MIA-PaCa2), prostate cancer (PC3), hepatocarcinoma (HepG2) (Fig. 1D)], and normal cells [normal human peripheral blood mononuclear cells (PBMC), mouse embryonic fibroblast cell line (NIH3T3), monkey kidney epithelial cell line (Vero) (Fig. 1E)]. Combination of HCH (10 µM) and BSO (100 µM) drastically reduced the viability of all the leukemic cell lines tested leaving other cancer cell lines and normal cells marginally affected. Also, HCH or BSO when tested alone, viability of all the cancer cell lines including leukemic cell lines and normal cells remained unaffected.

**Figure 1:** BSO potentiates HCH induced cytotoxicity in leukemic cells. (**A**) K562 cells were incubated with varying concentrations of HCH (left panel) and BSO (right panel) for 48 h and viability was determined by (3-(4,5-Dimethylthiazol-2-yl)-2,5-diphenyltetrazolium bromide (MTT) assay. Structures of HCH and BSO are shown within the respective graphs. * p<0.05 compared to treatment with vehicle control; ** p<0.01 compared to vehicle control. (**B**) K562 cells were simultaneously treated with varying concentration of BSO and HCH for 48 h. * p<0.05 compared to HCH treatment alone; ** p<0.01 compared to treatment with HCH alone; *** p<0.001 compared to HCH treatment alone; # p<0.01 compared to treatment with vehicle control or BSO. (**C**) Leukemic cell lines were incubated with BSO and HCH either alone or in combination for 48 h. *** p<0.001 compared to treatment with vehicle control or either of the compounds alone. (**D**) Same as (C) except that non-leukemic cancer cell lines were used instead of leukemic cell lines. (**E**) Normal cell lines or normal human peripheral blood mononuclear cells (hPBMC) were incubated with BSO and HCH either alone or in combination for 48 h. (**F**) PBMC from one normal donor and 3 CML patients were incubated with BSO and HCH either alone or in combination for indicated time periods and viability was determined by trypan blue dye exclusion assay. ** p<0.01 and *** p<0.001 compared to treatment with vehicle control or either of the compounds alone respectively. (A)-(F) Data represent mean ± SD of quadruplicate wells. (**G**) Isobologram analysis for the determination of synergy using Calcusyn software.

Preferential cytotoxicity of combination of low doses of HCH and BSO on leukemic cell lines prompted us to evaluate this combination on primary cells from three CML patients and one normal PBMC. Like leukemic cell lines, viability of all three CML patients’ PBMC was drastically reduced by the combination of BSO and HCH while viability of normal PBMC was marginally reduced (Fig. 1F). Isobologram analysis suggested that the cytotoxic effect of combination of HCH and BSO on K562 cells was synergistic (Fig. 1G).

### BSO Synergizes with HCH to Induce Apoptosis in a Time and Sequence Dependent Manner

The enhanced cytotoxic activity after combination of low doses of BSO and HCH against K562 cells was apoptotic in nature which was confirmed by flow cytometry after staining with annexin V and PI (Fig. 2A). The same combination had minimal effects on normal PBMC (Fig. 2B). However, apoptosis was undetectable when cells were treated with HCH, washed and then treated with BSO (Fig. 2C). In contrast, cytotoxicity was detectable when cells were treated with BSO first then washed and treatment with HCH followed (Fig. 2C). These data suggest that BSO sensitizes K562 cells to HCH- mediated apoptosis. Apoptosis was further supported by the decrease in mitochondrial membrane potential (Fig. S1A) and release of cytochrome c from mitochondria to cytosol (Fig. S1B).

**Figure 2:** Sequential administration of BSO potentiates HCH- induced apoptosis in caspase dependent manner. (**A**) K562 cells were treated with 100 µM BSO and 10 µM HCH either alone or in combination for indicated times and apoptosis was measured by annexin V/PI binding assay. Dot plots are representative of two similar experiments. (**B**) hPBMC were treated as indicated for 36 h and apoptosis was measured by annexin V/PI binding assay. Representative of two similar experiments. (**C**) BSO (100 µM) was administered 24 h prior addition of HCH (10 µM) and vice versa in K562 cells and incubated for 24 h for measurement of apoptosis by annexin V/PI binding assay. Representative of two similar experiments. (**D**) K562 cells were incubated with 100 µM BSO and 10 µM HCH or their combination for 24 h. Whole cell lysates were subjected to western blot analysis using indicated antibodies. Antibody to actin was used as loading control. (**E**) K562 cells were pre-treated with pan-caspase inhibitor Z-VAD-FMK (50 µM), caspase 8 inhibitor Z-IETD-FMK (50 µM) and caspase-9 inhibitor LEHD-CHO (25 µM) before treatment with BSO (100 µM) and HCH (10 µM). After 36 hours, cell viability was assessed using MTT assay. Every column represents mean ± SD of three experiments. *** p<0.001 compared to treatment with vehicle control; * p<0.05 compared to treatment with no caspase inhibitors.

### Combination of BSO and HCH-induced Apoptosis was Mediated by Caspase-dependent and Independent Pathways

Role of different caspases in apoptosis induced by combined treatment of BSO and HCH was then evaluated. Neither caspase-8 nor caspase-9 was cleaved by HCH or BSO alone or in combination (Fig. 2D). Significant cleavage of PARP and caspase-3 was noticed after combined treatment (Fig. 2D). These data are supported by performing cytotoxicity experiments in the presence of pharmacological inhibitors of different caspases. Pan caspase inhibitor (Z-VAD-FMK) partially reversed the cytotoxicity while inhibitor of caspase-8 or caspase-9 had no appreciable effects (Fig. 2E).

Only partial reversal of apoptosis of K562 cells in the presence of pan-caspase inhibitor suggested the possible role of caspase-independent process of apoptosis induced by combined treatment of HCH and BSO.

Apoptosis-inducing factor (AIF) is known to play an important role in caspase-independent apoptosis [30], [31]. We therefore evaluated activation of AIF after combined treatment of HCH and BSO. Translocation of AIF to nucleus in K562 cells was only detectable after combined treatment with BSO and HCH and as expected the nuclear translocation of AIF was unaffected in the presence of pan-caspase inhibitor (Fig. 3). Thus, our data suggest that apoptosis, induced in CML cells by combination of BSO and HCH, is executed by combination of caspase-dependent and –independent pathways.

**Figure 3:** Combination of BSO and HCH induces AIF translocation in caspase-independent manner. K562 cells were treated as indicated and processed for confocal microscopy as stated in Materials and Methods. Scale bar, 10 µm.

### Combination of HCH and BSO Causes Enhanced Depletion of Intracellular GSH in K562 Cells

BSO is a known depletor of intracellular GSH [32], [33]. HCH alone did not deplete intracellular GSH at a concentration of 10 µM (Fig. 4A). When HCH was combined with BSO, drastic depletion of intracellular GSH was noted in K562 cells in a time dependent manner (Fig. 4A). Of interest, the depletion of GSH was much higher in K562 cells compared to normal human peripheral blood mononuclear cells (Fig. 4B).

**Figure 4:** BSO potentiates HCH- induced apoptosis by depleting intracellular GSH. (**A**) K562 cells were treated as indicated for measurement of intracellular GSH as described in Materials and Methods. Data represent mean ± SD of three experiments. ** p<0.01 and *** p<0.001compared to treatment with BSO alone. (**B**) K562 cells and hPBMC were treated as indicated for 24 h and intracellular GSH was measured. Data represent mean ± SD of three experiments. # p<0.01 compared to vehicle control; ** p<0.01 compared to BSO alone. (**C)** K562 cells were treated as indicated for different time points and intracellular H_2_O_2_ were measured by flow cytometry after DCF-DA staining. Data represent mean ± SD of three experiments. ** p<0.01 compared to treatment with BSO or HCH alone. (**D**) K562 cells were preincubated with varying concentrations of glutathione monoethyle ester (GME) for 1 h and further incubated with BSO (100 µM) and HCH (10 µM) as indicated for 36 h. Percent apoptotic cells were calculated by flow cytometry after annexinV-PI staining. Data represent mean of three experiments. ** p<0.01 compared to treatment in absence of GME. *** p<0.001 compared to treatment in absence of GME. (**E**) K562 cells were pre-incubated with 2 mM GME for 1 h and further incubated with BSO (100 µM) and HCH (10 µM) in combination for 36 h. Mitochondrial membrane potential was assessed in a flow cytometer after staining with JC-1 dye. Dot plots and histograms are representative of two similar experiments.

### Combination of HCH and BSO Causes Enhanced Production of ROS

Enhanced intracellular ROS was detectable in K562 cells only in the presence of HCH plus BSO and this was detectable at 4 h onwards (Fig. 4C). Time kinetics of depletion of intracellular GSH correlates with that of detection of intracellular ROS. These data suggest that enhanced depletion of intracellular GSH may be responsible for production of enhanced ROS in the presence of BSO plus HCH. Apoptosis of K562 cells induced by the treatment of BSO plus HCH was completely reversed by pretreatment with glutathione precursor glutathione monoethyle ester (GME) in a dose dependent manner (Fig. 4D), suggesting the role of glutathione depletion in BSO plus HCH-induced ROS production and apoptosis. BSO plus HCH-induced decrease in mitochondrial membrane potential and release of cytochrome c from mitochondria was also reversed by GME (Fig. 4E, Fig. S1C).

### Combination of HCH and BSO Causes Enhanced Production of Nitric oxide (NO)

Intracellular NO was detectable in K562 cells in the combined presence of HCH and BSO no earlier than 18 h which was further increased in a time dependent manner (Fig. 5A). Increase of intracellular NO was also detectable in normal hPBMC, however, this was significantly lower than that observed in K562 cells (fold increase of NO in hPBMC was 1.3 vs. 3.3 in K562 cells under the same experimental condition) (Fig. 5B). Next we evaluated the effect of nitric oxide scavenger (cPTIO) on HCH plus BSO-mediated apoptosis of K562 cells. As shown in Fig. 5C, cPTIO not only scavenged HCH plus BSO-induced NO (right panel) but also reversed the apoptosis (left panel). Cleavage of PARP and caspase-3 was also inhibited in the presence of cPTIO (Fig. 5D). Combination of HCH and BSO induced ROS production detectable as early as 4 h whereas induction of NO by the same combination was detectable only after 18 h. We therefore evaluated whether production of NO was dependent of ROS production or independent of ROS. As shown in Fig. 5E, HCH plus BSO-induced NO production was completely inhibited when K562 cells were pre-incubated with ROS scavenger GME. Therefore, NO produced in K562 cells by the combined treatment of HCH and BSO were solely dependent on early production of ROS.

**Figure 5:** Combination of BSO and HCH induces NO production in CML cells that causes apoptosis. (**A**) K562 cells were treated as indicated for different time periods and then intracellular nitric oxide (NO) was measured by flow cytometry after staining with DAF-FM. Data represent mean ± SD of three experiments. ** p<0.01 compared to treatment with either BSO or HCH alone. *** p<0.001 compared to treatment with either BSO or HCH alone. (**B**) Representative histograms of DAF-FM staining in K562 cells and hPBMC after treatment as indicated for 24 h. (**C**) K562 cells were pretreated with 100 µM cPTIO for 2 h followed by incubation with combination of 100 µM BSO and 10 µM HCH for 24 h. Cells were then subjected to annexin V/PI binding assay by flow cytometry (left panel). Histograms show measurement of NO in the presence or absence of cPTIO after indicated treatment (right panel). Representative of two similar experiments. (**D**) K562 cells were treated as indicated for 24 hours after pretreatment with 100 µM cPTIO for 2 h. The whole cell lysates were then immunoblotted with indicated antibodies. (**E**) K562 cells were pre-incubated with indicated concentrations of GME followed by treatment with BSO and HCH as indicated for 24 h. Analysis of intracellular NO was done by flow cytometry after staining with DAF-FM. Histograms are representative of two similar experiments.

### Combination of HCH and BSO Activates JNK and ERK Pathways: JNK Positively Regulates ERK

JNK and ERK have been reported to be involved in NO production through the activation of nitric oxide synthase enzyme [29], [34]. We therefore tested the phosphorylation of MAP kinases in the presence of HCH, BSO and HCH plus BSO. Neither HCH nor BSO at the low doses tested, induced phosphorylation of JNK, ERK or p38. However, phosphorylation of JNK was detectable at 6 h while that of ERK started appearing at 12 h when HCH and BSO were combined (Fig. 6A). Phospho-p38 remained undetectable throughout the incubation period of 24 h (Fig. 6A). Of note, apoptotic dose of HCH alone induced JNK phosphorylation only (Fig. S2); [16]. Role of JNK and ERK in HCH plus BSO-mediated apoptosis of K562 cells was then evaluated by (i) using pharmacological inhibitors and (ii) knocking down these MAPKs using specific siRNAs. Pharmacological inhibitor of p38 MAPK had no appreciable effects on HCH plus BSO-mediated apoptosis of K562 cells while pre-incubation with inhibitor of JNK or ERK significantly reversed the apoptosis (Fig. 6B). These data were further supported by knockdown experiments where JNK1 or ERK2 proteins were knocked down in K562 cells using specific siRNAs before treatment with HCH plus BSO (Figs. 6C, 6D). Two scrambled sequences of siRNA which did not have sequence similarity to either JNK or ERK mRNA were used as controls. Therefore, both MAPKs JNK and ERK played important role in HCH plus BSO-mediated apoptosis.

**Figure 6:** Apoptosis induced by combination of BSO and HCH is mediated by JNK dependent ERK1/2 activation. (**A**) K562 cells were treated as indicated for different time periods and cell lysates were subjected to western blot analysis with indicated antibodies. (**B**) K562 cells were pretreated with JNK inhibitor SP600125 (20 µM), p38 inhibitor SB203580 (20 µM), ERK inhibitor PD98059 (40 µM) for 1 h before treatment with BSO (100 µM) and HCH (10 µM) in combination. After 36 h of incubation, cells were subjected to Annexin V/PI binding assay by flow cytometry. Data represent mean ± SD of three experiments. *** p<0.001 compared to treatment in absence of MAPK inhibitors. (**C**) Knockdown of JNK by specific JNK1 siRNA attenuates apoptosis. JNK1 protein level was shown after knockdown (upper panel). Annexin V/PI binding assay by flow cytometry in K562 cells after transfection with indicated siRNAs (lower panel). Dot plots are representative of two similar experiments. (**D**) Knockdown of ERK by specific ERK2 siRNA attenuates apoptosis. ERK2 protein level was shown after knockdown (upper panel). Annexin V/PI binding assay by flow cytometry after knocking down ERK2 (lower panel). Dot plots are representative of two similar experiments (**E**) K562 cells were transfected with indicated siRNAs for 48 h and then treated with BSO plus HCH for 18 h. Protein expression and phosphorylation of JNK and ERK1/2 were analysed by western blot on whole cell lysates. (**F**) K562 cells were pre-incubated with or without 2 mM GME for 1 h and further incubated with BSO (100 µM) and HCH (10 µM) in combination for 18 h. The level of each protein and phosphorylation status was analyzed as indicated by western blot. (**G**) K562 cells were transfected with indicated siRNAs for 48 h and then treated with BSO plus HCH for 24 h. Analysis of intracellular NO was done by flow cytometry after staining with DAF-FM. Histograms are representative of two similar experiments.

We next evaluated the possible crosstalk between JNK and ERK in HCH plus BSO-mediated apoptosis of K562 cells, keeping in mind that JNK negatively regulates ERK activity [35], [36], [37]. Western blot analysis indicate that knocking down JNK1 reduced phosphorylation of ERK in K562 cells while knocking down ERK2, phosphorylation of JNK remained unaffected (Fig. 6E). Activation of both JNK and ERK was dependent on HCH plus BSO-mediated ROS production as pretreatment of K562 cells with ROS scavenger GME before the combined treatment completely reversed the phosphorylation of both the MAPKs (Fig. 6F).

### HCH Plus BSO-mediated NO Production Comes from Inducible Nitric Oxide Synthase (iNOS) and Dependent on JNK or ERK Activation

Knocking down ERK2 or JNK1 from K562 cells significantly reduced HCH plus BSO-mediated NO production (Fig. 6G), suggesting the role of these MAPKs in NO production. We next tried to identify the isoform of NOS in K562 cells producing NO in the presence of HCH plus BSO. Time kinetics of the protein expression and phosphorylation status of the NOS isoforms in K562 cells after treatment with HCH, BSO or combination of both suggest that treatment with HCH plus BSO increased the expression of iNOS protein without affecting eNOS or nNOS neither at the level of protein expression nor at the level of phosphorylation (Fig. 7A). To evaluate whether HCH plus BSO-mediated NO production in K562 cells was coming from iNOS, knockdown experiments were performed in K562 cells with isoform-specific siRNAs before evaluation of NO production. Knocking down iNOS reduced the level of intracellular NO while transfection with eNOS or nNOS siRNA had no effects (Fig. 7B). Transfection with specific siRNAs yielded reasonable knockdown of the respective isoforms (Fig. 7C). Similarly, apoptosis was also mostly reversed by knocking down iNOS only (Fig. 7D) and activation of iNOS expression was dependent on both JNK and ERK (Fig. 7E). However, activation of JNK or ERK was independent of iNOS expression (Fig. 7F), suggesting that iNOS is downstream of JNK or ERK. So far we demonstrated that scavenging ROS reversed BSO plus HCH-mediated apoptosis of K562 cells and apoptosis is mostly mediated by ROS-dependent activation of JNK and ERK leading to activation of iNOS expression. iNOS- mediated production of NO was identified as the key effector molecule of apoptosis. This is further supported by Fig. 7G which indicates that scavenging ROS reverses iNOS expression while knocking down iNOS failed to restore depleted intracellular glutathione (Fig. 7H).

**Figure 7:** Nitric oxide is produced by inducible nitric oxide synthase (iNOS); iNOS expression is dependent on ERK 1/2 and JNK activation. (**A**) K562 cells were treated as indicated for varying time periods and the whole cell lysates were subjected to western blot analysis with indicated antibodies. (**B**) After transfection of K562 cells with indicated siRNAs followed by indicated treatments for 24 h, cells were stained with DAF-FM for measurement of NO. Representative of two similar histograms. (**C**) K562 cells were transfected with control siRNA or indicated NOS siRNAs for 48 h and then treated with combination of BSO (100 µM) and HCH (10 µM) for 24 h. Whole cell lysates were subjected to western blot for the expression of indicated proteins to confirm knockdown of representative NOS isoforms. (**D**) K562 cells were subjected to annexin V/PI binding assay by flow cytometry after 36 h. Representative of two similar histograms. (**E**) K562 cells were transfected with JNK1 or ERK2 siRNA. Cells were then treated with combination of BSO (100 µM) and HCH (10 µM) for 18 h. Cell lysates were then immunoblotted with anti-iNOS antibody. (**F**) iNOS siRNA transfected K562 cells were treated with combination of BSO (100 µM) and HCH (10µM) for 18 h and subjected to immunoblot analysis with indicated antibodies. (**G**) K562 cells were pre-incubated with GME for 1 h before treatment with combination of BSO and HCH for 18 h and cell lysates were then immunoblotted with anti-iNOS antibody. (**H**) GSH measurement was done in iNOS transfected K562 cells after combined treatment with BSO and HCH for 18 h. Data represent mean ± SD of three experiments. *** p<0.001 compared to vehicle control.

## Discussion

Cancer cells have long been known to have higher oxidative stress than their normal counterparts. Manipulation of intracellular oxidative stress either by antioxidants [38] or by pro-oxidants [39], [40] have also been exploited for preferential killing of cancer cells. We recently reported that hydroxychavicol purified from *Piper betle* leaves or prepared synthetically induces apoptosis of CML cells by ROS-dependent JNK- mediated eNOS activation and IC50 for K562 cells was more than 20.0 µM [16]. Depletion of intracellular GSH might potentiate intracellular threshold of ROS and had also been exploited for cancer cell killing [41], [42]. Disruption of the intracellular redox state by altered GSH content affects the activation signaling pathways, which could make cancer cells susceptible to toxic insults. GSH is known to fulfill multiple defensive functions in the cell [43]. It represents an essential component of the detoxification machinery, which rids the cells of pharmacologic drugs and other toxicants. BSO is one such agent which depletes intracellular GSH by inhibiting gamma-glutamylcysteine synthetase [3]. In the present study we evaluated the effect of combination of low doses of HCH and BSO on the cytotoxicity on a number of leukemic and non-leukemic cancer cell lines as well as primary cells from normal donors and CML patients. The combination is also effective on primary cells from CML patients. Of note, cancer cell lines of other origin like lung, prostate, pancreas, liver and a number of normal cell lines and normal human peripheral blood mononuclear cells were less affected by the combination.

We attempted to elucidate the mechanism of BSO plus HCH-induced apoptosis in CML cells. We observed that BSO and HCH in combination induced apoptosis in a time-dependent manner in K562 cells. We found that the combination activated caspase-3 and PARP. Pre-treatment of the cells with Z-VAD-FMK partially blocked BSO and HCH-induced cell death. These results suggested that BSO plus HCH-induced apoptosis in CML cells may not fully dependent on caspase activation. It has been reported that AIF-mediated apoptosis is a caspase-independent event. Confocal microscopy study revealed translocation of AIF to nucleus which were not inhibited by Z-VAD-FMK. This result suggested the activation of AIF in caspase-independent manner.

Here, we demonstrated an inverse correlation between cellular GSH levels and HCH sensitivity of CML cells. We established that co-treatment with BSO enhanced the cytotoxicity of HCH in CML cells. With BSO, low concentrations of HCH depleted intracellular GSH levels and resulted in an increase in CML cells apoptosis. Combining low doses of HCH and BSO drastically potentiated the depletion of intracellular GSH from CML cells leading to generation of ROS. HCH alone at this non-apoptotic concentration did not deplete intracellular GSH although BSO alone causes detectable depletion, however, to a significantly lesser extent than the combination. The exact mechanism that leads to enhanced depletion of GSH from CML cells by combination of BSO and HCH is yet to be determined and also reason for lower depletion of GSH from normal hPBMC even in the presence of combined treatment is not clear.

As mitogen-activated protein kinases (MAPKs) are involved in stress induced apoptosis, we evaluated the role of MAPKs in this BSO plus HCH mediated signaling cascade. HCH-induced apoptosis included activation of JNK and p38 kinase without any role of ERK [16]. The combined treatment led to activation of both JNK and ERK1/2. The activatory phosphorylation of JNK was detected earlier than ERK1/2. As JNK and ERK1/2 were activated in a sequential manner we evaluated their cross talk. Knockdown experiments established that JNK is activating ERK1/2 but ERK1/2 had no effect on JNK activation. Thus early and sustained activation of JNK is activating ERK1/2 and not the vice versa. The cross talk between JNK and ERK has been reported earlier. Some of the reports suggested negative regulation of ERK by JNK [35], [37], [44] **.** Other reports suggested independent activation of these MAPKs in apoptotic event [20], [29]. Here we report for the first time that JNK positively regulated ERK leading to apoptosis of CML cells.

The GSH depletion was the earliest event in BSO plus HCH-induced signaling and the apoptotic effect of this combination was correlated with the enhanced depletion of GSH as glutathione precursor GME abrogated activation of JNK, ERK and the apoptosis.

Several studies established nitric oxide as an effector of apoptosis [45], [46]. Our study showed that BSO plus HCH-induced apoptosis involved the generation of reactive nitrogen species and nitric oxide scavenger cPTIO partially but significantly blocked the apoptosis induction and NO formation. However, the reversal of apoptosis was only around 30%. This is probably because of incomplete scavenging of NO by cPTIO. The residual NO may have caused the detectable apoptosis even in the presence of cPTIO. Higher concentration of cPTIO could not be used in apoptosis- reversal experiment because of toxicity induced by cPTIO itself. Activation of cleaved form of caspase 3 and PARP was also partially blocked by cPTIO suggesting the role of NO in apoptosis. siRNA of either JNK or ERK successfully blocked the production of NO, the expression of iNOS and apoptosis. The role of NO in combined treatment- induced apoptosis is further supported by the knock down experiment with siRNA of iNOS. Reversal of apoptosis by knocking down iNOS was comparable to that of JNK or ERK knock down. iNOS knockdown revealed that although iNOS had no effect on the activation of JNK and ERK1/2 and GSH depletion, it played important role in apoptosis.

iNOS overexpression or iNOS inducer has apoptotic effects on cells. LPS- mediated iNOS induction caused apoptosis in endothelial cells [47], in murine macrophage-derived RAW cells [48] and in cardiac myocytes [49]. Similarly, transfection or overexpression of iNOS causes apoptosis in vascular smooth muscle cells [50] or suppresses the tumorigenicity and metastasis of oral cancer cells [51].

However, restoration of intracellular GSH level inhibited the expression of iNOS. Thus, GSH depletion by combination of BSO and HCH resulted in increased production of NO by iNOS through the activation of JNK mediated ERK pathway leading to apoptosis of CML cells.

In conclusion, the present study demonstrates a potent anti-CML activity of the combination of BSO and HCH in vitro and elucidates the molecular mechanisms, which are dependent on GSH depletion. Our study also established JNK as a positive upstream regulator of ERK1/2. It is, therefore, possible that such combination therapy may provide a potential strategy for increasing the efficacy of traditional chemotherapeutics in killing CML cells.

## Supporting Information

Figure S1 **BSO potentiates HCH- mediated mitochondrial membrane potential disruption and cytochrome c release. (A)** K562 cells were treated as indicated for 24 hours. The cells were stained with JC-1 dye and subjected to flow cytometry. Representative of two similar experiments. **(B)** Cell lysates were subjected to western blot for cytochrome c. **(C)** K562 cells were pretreated with GME (2 mM) for 1 hour followed by treatment with BSO and HCH as indicated. Whole cell lysates were subjected to western blot analysis for cytochrome c.
(TIF)

Figure S2 **HCH activates JNK not ERK.** K562 cells were incubated with HCH for different time points. Whole cell lysates were immunoblotted with indicated antibodies.
(TIF)
